# Application Effect of the 6S Care Model in Sterilization in the Department of Stomatology and Its Impact on the Incidence of Nosocomial Infection

**DOI:** 10.1155/2022/4266087

**Published:** 2022-07-18

**Authors:** Jing Lou, Guiqin Wang, Man Jiang, Guochao Xu

**Affiliations:** Department of Stomatology, Affiliated Zhejiang Hospital, Zhejiang University School of Medicine, Hangzhou, Zhejiang 310013, China

## Abstract

**Objective:**

The study aimed to explore the effectiveness of the 6S care model in sterilization in department of stomatology and its impact on the incidence of nosocomial infections.

**Methods:**

The infection surveillance indicators of the department of stomatology implementing the routine sterilization care model in 2019 were selected as the general group (including 140 patients and 140 cases of oral instrument kits for unpacking), and the infection surveillance indicators of the department of stomatology implementing the 6S care model in 2020 were selected as the 6S group (including 140 patients and 140 cases of oral instrument kits for unpacking). Analysis of the air culture qualification rate of the consultation room + operating room, medical equipment sterilization qualification rate, medical equipment damage rate, incidence of nosocomial infections, satisfaction of medical and nursing staff with instrument sterilization, and patient satisfaction with medical and nursing staff care services under different care models was carried out.

**Result:**

The air culture pass rate of the consultation room + operating room in the 6S group was 96.43% (135/140), which was higher than 90.00% (126/140) in the general group, and the difference between the two groups was statistically significant (*P* > 0.05). The sterilization pass rate of medical devices in the 6S group was 100% (140/140), which was higher than 95.71% (134/140) in the general group, and the difference between the two groups was statistically significant (*P* > 0.05). The medical device damage rate in the 6S group was 0.71% (1/140), which was lower than 7.14% (10/140) in the general group, and the difference between the two groups was statistically significant (*P* > 0.05). The incidence of nosocomial infection in the 6S group was 0.71% (1/140), lower than 5.71% (8/140) in the general group, and the difference between the two groups was statistically significant (*P* > 0.05). In the 6S care model, the satisfaction score of 38 healthcare workers with the disinfection of instruments was (96.55 ± 2.40), which was higher than that of the general group (87.79 ± 3.14), and the difference between the two groups was statistically significant (*P* > 0.05). The total nursing satisfaction of the 6S group was 97.86% (137/140), which was higher than 91.43% (128/140) of the general group, and the difference between the two groups was statistically significant (*P* > 0.05).

**Conclusion:**

The application of the 6S care model in the sterilization of the department of stomatology can significantly improve the passing rate of infection monitoring indicators in the department of stomatology, reduce the occurrence of medical device damage and nosocomial infection, and have high satisfaction among doctors and patients, which has the value of promotion.

## 1. Introduction

The diversification of dental services has led to an increase in the range of dental instruments involved, but with this comes the problem of nosocomial infections in the department of stomatology [1, 2]. For example, when the cleaning and disinfection of oral instruments are unqualified, residual organic matter can form a protective film on the surface of the instrument, and pathogens and other microorganisms grow in the protective film. When the instrument is applied to patients with oral diseases, microorganisms take the opportunity to invade the oral cavity, causing nosocomial infection and increasing medical disputes [3]. In addition, the oral cavity, as the beginning of the gastrointestinal and respiratory tracts, has long been in contact with the outside world and is itself a place where bacteria can collect and breed, so when traumatic operations are performed on patients in the oral cavity, residual germs can easily colonise the mouth and cause infections in the surgical wound, gastrointestinal tract, or respiratory tract [4, 5]. Therefore, strict enhancement of sterile care management in the department of stomatology is of great significance in reducing the risk of oral infections after treatment, facilitating patients' prognosis for recovery and reducing the risk of nosocomial cross infection in the department of stomatology.

The 6S nursing model originated in Japan and consists of six elements: “seiri, seiton, seiso, seiketsu, shitsuke, and safety.” It is a systematic management model used in operating theatres, wards, and outpatient clinics [6, 7]. Its emphasis on improving the quality of care and reducing nosocomial infections through behavioural management and site tidying and cleaning is centred on improving the professionalism of medical staff. However, the effectiveness of its implementation and impact on the occurrence of nosocomial infections when applied to sterilization management in the department of stomatology has been less reported. In this study, the infection surveillance indicators of the department of stomatology without the implementation of the 6S care model in 2019 were used as a control to analyse the effect of the application of the 6S care model in the disinfection of the department of stomatology and the impact on the incidence of nosocomial infections since 2020. This is reported in the following sections.

## 2. Materials and Methods

### 2.1. General Data

The study was carried out by 25 dentists, 5 nurses, and 8 assistants in 33 consultation rooms and 2 operating theatres in our department. A convenience sampling method was used to select 140 patients and 140 oral instrument kits used in each of the 2019 and 2020 periods for infection surveillance indicators. The infection surveillance indicators of the department of stomatology implementing the routine sterile care model in 2019 were used as the general group, and the infection surveillance indicators of the department of stomatology implementing the 6S care model in 2020 were used as the 6S group.

### 2.2. Nursing Mode

#### 2.2.1. The General Group Implemented a Routine Sterile Care Model

(1) To establish and improve various aseptic sterilization systems, such as norms for the use of disposable medical items, dedicated management of dental drugs, hand hygiene system, centralised sentinel sterilization management of dental instruments and tools, air disinfection system in dental consultation rooms, and medical waste management should be followed. (2) To strengthen disinfection and sterilization management, medical personnel should carry out dental treatment operations under the condition of wearing protective gear, operate according to standard procedures, avoid occupational exposure, wash hands, and disinfect strictly before and after each operation; if the treatment chair or lights needed to be readjusted during the treatment process, the nurse should cooperate with the adjustment, and the operating physician should be strictly prohibited from touching surrounding objects with contaminated hands. Disinfection of dental instruments should be in the order of “decontamination, cleaning, and sterilization.” Disinfection of dental equipment should be in the “disinfection, cleaning, and sterilization” sequence. Regular disinfection of the environment and air in consultation rooms and operating theatres should be performed. (3) Medical waste was managed separately, and these were registered and handed over daily and recorded and filed.

#### 2.2.2. The Experimental Group Implemented the 6S Care Model

(1) For launching the 6S nursing management conference, the participants were all the medical staff of the department of stomatology. The conference included an introduction to the background, requirements, and objectives of 6S implementation, an announcement of the 6S committee's organisational structure and responsibilities, 6S implementation methods and schedule, 6S inspection standards and audit and evaluation programmes, and an oath for 6S committee members. (2) The nosocomial infection prevention and control team was established in the department with the head nurse as the team leader to coordinate site management, disinfection of items, training, and appraisal. (3) To develop 6S nursing management standards, the prevention and control team shall develop systems and annual management KPIs (key performance indicators) related to nosocomial infection protection. For example, sterilization norms for instruments, management of sterile items, hand hygiene and the surface cleaning system for items, air disinfection system, material collection and management, medical waste management system, and training and assessment system should be followed. The implementation targets were for team members to be familiar with the knowledge and skills within 1 month and to be fully competent and flexible in applying the knowledge and skills within 2 months. (4) To implement and monitor the 6S care system, systematic training, daily supervision, and assessment should be performed. The management team carefully completed the learning and training of relevant knowledge and its skills to ensure that everyone mastered and passed the assessment. The training covered precautions related to infection prevention, aseptic practices, procedures, and methods. This training also covered the cleaning staff in the hospital. In addition, healthcare workers should pay attention to the cleaning and disinfection of hands, ensuring that they always “disinfect after use” and “disinfect after treatment.” In outpatient site management, all types of dental items should be sorted and discharged in an orderly manner, and medical waste after dental treatment should be cleaned up in a timely manner. In item management, medical supplies were entered into the system, sterilized items were sorted into categories and placed according to sterilization expiry dates, and the computer system automatically displayed the sterilization expiry dates. In addition, cleaners were required to place cleaning tools (mops, rags, etc.) in a fixed location according to their function and area of use, and mixing them was strictly prohibited. (5) Group members gave weekly feedback on their own hygiene management and set up 6S hygiene management Kanban boards, and each person must update their respective Kanban records daily. All group members were assessed once a month and the assessment results were linked to performance.

### 2.3. Evaluation Indicators

1. Passing of the air culture: We compared the passing of the air culture in the consultation room + operating room in 140 cases each in the 6S group and the general group.
2. Evaluation of the sterilization effect of medical devices: the disinfection effect of 140 cases of dental instrument kits that were disinfected after opening and being used during 2019 and 2020 was evaluated according to the “Hospital Disinfection Hygiene Standards” (GB15982-2012) [8] promulgated by the Ministry of Health in 2012. A cotton swab soaked in sterile saline sampling solution was applied to the surface of the instrument for sampling. The finished swab was placed in a test tube containing the sampling solution, and the sample was cultured for bacteria using the agarose culture method. A positive sample with colony growth was considered to have failed sterilization, and a negative sample with no colony growth was considered to have passed sterilization.
3. Damage to medical equipment: we compared the damage to dental medical equipment in 140 cases each in the 6S group and the general group.
4. Incidence of nosocomial infections: the diagnostic criteria for nosocomial infections were based on the “Diagnostic Criteria for Hospital Infections” [9] issued by the Ministry of Health in 2001. The number of cases of nosocomial infections in each of the 140 patients in the 6S and general groups was compared.
5. Healthcare workers' satisfaction with instrument sterilization: the survey scale was self-made within the department. A total of 25 items, each with a score of 0 to 4 out of 100, were used to compare the satisfaction scores of 38 healthcare professionals in the department of stomatology with regard to the sterilization of instruments. Higher scores indicated that patients were more satisfied with the quality of disinfection of the instruments.
6. Patient satisfaction with care it was evaluated by patients completing a care satisfaction questionnaire. The questionnaire was self-administered within the department and had a 3-point scale, with 3 points for very satisfied, 2 points for satisfied, and 0 point for dissatisfied, for a total of 16 items. The cumulative total rough score for each item was 48, with scores of 0–28 being dissatisfied, 29–38 being satisfied, and 39–48 being very satisfied. Total satisfaction = (very satisfied + satisfied)/total number of cases × 100%. This formula was used to compare the satisfaction ratings of 140 patients in each of the 6S group and the general group with regard to the nursing services provided by the healthcare staff.

### 2.4. Statistical Methods

Data analysis was processed by SPSS 22.0 software. The count data were expressed as (%), and the *χ*^2^-test analysis was used for comparison. The measurement data were expressed as ($\bar{x}\pm s$), and the *t*-test analysis was used for comparison. *P* < 0.05 indicated that the difference was statistically significant.

## 3. Results

### 3.1. Analysis of Air Culture Compliance in Two Groups of Consultation Rooms + Operating Rooms

The air culture pass rate of the consultation room + operating room in the 6S group was 96.43% (135/140), which was higher than 90.00% (126/140) in the general group, and the difference between the two groups was statistically significant (*P* > 0.05) as seen in Figure 1.

### 3.2. Analysis of the Disinfection Effect of Dental Medical Devices in Two Groups

The sterilization pass rate of medical devices in the 6S group was 100% (140/140), which was higher than 95.71% (134/140) in the general group, and the difference between the two groups was statistically significant (*P* > 0.05) as seen in Figure 2.

### 3.3. Analysis of Damage to Medical Devices in Two Groups of Dentists

The medical device damage rate in the 6S group was 0.71% (1/140), which was lower than 7.14% (10/140) in the general group, and the difference between the two groups was statistically significant (*P* > 0.05) as seen in Figure 3.

### 3.4. Analysis of Nosocomial Infections in Two Groups of Patients

The incidence of nosocomial infection in the 6S group was 0.71% (1/140), which was lower than 5.71% (8/140) in the general group, and the difference between the two groups was statistically significant (*P* > 0.05) as seen in Figure 4.

### 3.5. Analysis of the Satisfaction of 38 HealthCare Workers with the Sterilization of Instruments

In the 6S care model, the satisfaction score of 38 healthcare workers with the disinfection of instruments was (96.55 ± 2.40), which was higher than that of the general group (87.79 ± 3.14), and the difference between the two groups was statistically significant (*P* > 0.05) as seen in Figure 5.

### 3.6. Analysis of Patient Satisfaction with Care in Both Groups

The total nursing satisfaction of the 6S group was 97.86% (137/140), which was higher than 91.43% (128/140) of the general group, and the difference between the two groups was statistically significant (*P* > 0.05) as seen in Figure 6.

## 4. Discussion

Nosocomial infection, as an important indicator of the level of hospital management and the quality of management, is a constraint on the standard of care. The stomatology department is a high-risk department for nosocomial infections because of its complex treatment environment, high staff mobility, small and precise instruments, complex structure, and frequent use, and tendency to breed and multiply bacterial microorganisms [10–12]. Therefore, it is necessary to strictly control the quality standard of infection prevention and control in the hospital and to manage the related prevention and control. The “6S” management, which originated from the modern Japanese corporate management, consists of six elements: seiri, seiton, seiso, seiketsu, shitsuke, and safety. Seiri, i.e., keeping everything in its place and removing what is unnecessary. Seiton, i.e., the rational arrangement of useful items, sorted, and organised. Seiso, i.e., cleaning the working environment and keeping it clean and tidy. Seiketsu, i.e., maintaining the results of organising, tidying and cleaning, and standardizing, and institutionalising their practice. Shitsuke i.e. taking human nature as a starting point and striving to improve the quality of all staff through the fact of tidying up and cleaning up. Safety, i.e., removing all possible unsafe elements [13]. This management model leads to an overall improvement in the quality of management and to the improvement and refinement of the quality system.

The monitoring of nosocomial infection indicators is an important tool for the prevention and control of hospital-acquired infections and can be used to reflect the current status of prevention and control of hospital-acquired infections and their management in a timely manner. Environmental hygiene indicators include monitoring of air, object surfaces, and hand hygiene of healthcare workers [14–16]. In this result, the air culture pass rate and medical device sterilization pass rate of the 6S group were higher than those of the general group, and the medical device damage rate and the incidence of nosocomial infection of the 6S group were lower than those of the general group (*P* > 0.05). The possible reasons for the analysis are the following: firstly, a well-organised nosocomial infection management in the department of stomatology can avoid nosocomial cross infection in addition to providing a clean, tidy, aesthetically pleasing, and safe treatment environment [17]. Secondly, assessment and satisfaction evaluation of healthcare workers' working conditions, especially linked to their performance can motivate healthcare workers to do their jobs better and more effectively and reduce errors in their work [18, 19]. Thirdly, the training of the whole staff to improve the professional nursing knowledge and competence of the medical and nursing staff will help to continuously improve the operation process and the standardization of the operation and enhance the professionalism. Therefore, the application of the 6S care model in the management of nosocomial infections in the department of stomatology has some value for promotion. The results of this study also showed that in the 6S care model, 38 healthcare workers rated their satisfaction with the sterilization of instruments higher than the general group, and the 6S group had higher total satisfaction with care than the general group (*P* > 0.05). This may be due to the fact that this study is based on the original management content of the hospital to regulate the work content of organising and cleaning, which, on the one hand, makes the process of cleaning and disinfection of medical devices in the hospital more standardized and ensures the safe use of dental instruments and medical safety; On the other hand, strengthening the hand hygiene of healthcare workers and reducing contact with pathogenic bacteria and airborne problems will not only provide a better and safer treatment environment for patients and avoid related medical disputes but also reduce the damage caused to instruments by the adhesion of organic materials, indirectly improving patient satisfaction with the use of dental instruments.

This study applied the 6S care model to the sterilization management of the stomatology department, which was widely recognized by the hospital leadership and also received strong support from the medical staff in the department. Both the initial mobilization meeting and the subsequent training activities provide guidance to dental medical workers from an intuitive and convenient perspective. This not only restrains the work behaviour of the medical staff and improves their poor work habits but also allows for timely correction of misconceptions in the workplace through communication and exchange between medical staff, which increases their knowledge of infection and leads to better infection prevention and control, avoiding adverse events and thus ensuring medical safety.

To sum up, the application of the 6S care model in the sterilization of the department of stomatology can significantly improve the passing rate of infection monitoring indicators in the department of stomatology, reduce the occurrence of medical device damage and nosocomial infection, and have high satisfaction of doctors and patients, which has the value of promotion.

## Figures and Tables

**Figure 1:** Analysis of air culture compliance in two groups of the consultation rooms + operating rooms. (a) Status of the qualified rate of air culture in clinic (cases). (b) The qualified rate of air culture in clinic (%). The 6S group compared to the general group, ^*∗*^*P* > 0.05.

**Figure 2:** Analysis of the disinfection effect of dental medical devices in two groups. (a) Disinfection effect (cases). (b) Sterilization qualification rate (%). The 6S group compared to the general group, ^*∗*^*P* > 0.05.

**Figure 3:** Analysis of damage to medical devices in two groups of dentists. (a) The damaged status of medical devices (cases). (b) Damage rate (%). The 6S group compared to the general group, ^*∗*^*P* > 0.05.

**Figure 4:** Analysis of nosocomial infections in two groups of patients. (a) The status of nosocomial infections (cases). (b) The incidence of nosocomial infections (%). The 6S group compared to the general group, ^*∗*^*P* > 0.05.

**Figure 5:** Analysis of the satisfaction of 38 healthcare workers with the sterilization of instruments. (a) Satisfaction score (scores). (b) Satisfaction score (scores). The 6S group compared to the general group, ^*∗*^*P* > 0.05.

**Figure 6:** Analysis of patient satisfaction with care in both groups. (a) Satisfaction score (scores). (b) Total nursing satisfaction (%). The 6S group compared to the general group, ^*∗*^*P* > 0.05.

## Data Availability

The primary data to support the results of this study are available upon reasonable request from the corresponding author.
